# Gastrokine 2 Regulates the Antitumor Effect of JAK2/STAT3 Pathway in Gastric Cancer

This article has been retracted.

**DOI:** 10.1155/2021/1343808

**Published:** 2021-08-02

**Authors:** Yu Zhou, Shan Xu, Jiao Liu, Yaping Zhu, Yaxin Zhu, Wei Li, Hui Ling

**Affiliations:** ^1^The First Affiliated Hospital of Shaoyang University, Shaoyang, Hunan 422000, China; ^2^Shaoyang University, Shaoyang, Hunan 422000, China; ^3^Key Laboratory of Tumor Cellular & Molecular Pathology (University of South China), College of Hunan Province, Cancer Research Institute, Hengyang Medical College, University of South China, Hengyang, Hunan 421001, China; ^4^Department of Pathology, Changsha Fourth People's Hospital, Changsha, Hunan 410006, China

## Abstract

GKN2 (gastrokine 2) mainly plays a regulatory role in gastric mucosal defense and cell protection mechanisms, and its role in gastric cancer has not been thoroughly elucidated. Immunohistochemistry was used to detect GKN2 and TFF1 expressions in 90 gastric cancer tissues, 48 neoplastic resection margins, and 22 normal gastric mucosa epithelia. It showed that the downregulation of GKN2 and TFF1 expressions in gastric cancer tissues was significantly different from that in adjacent normal gastric tissues and distal gastric mucosal tissues. Nevertheless, correlation analysis showed that GKN2 expression in gastric cancer tissues was independent of TFF1 expression. After overexpression of GKN2 was constructed in human gastric cancer cell line MKN28 with the Ad-GFP-GKN2 transfected, cell viability was measured by CCK-8 assay, and migration and invasion ability were analyzed by transwell migration assay and transwell invasion assay. It indicated that overexpression of GKN2 significantly reduced the viability of MKN28 and SGC7901 cells. Overexpression of GKN2 could also inhibit the migration and invasion ability in MKN28 and SGC7901 cells. In addition, upregulation of GKN2 can inactivate the JAK2/STAT3 pathway. Our data suggest that GKN2 and TFF1 play the antitumor role in gastric carcinoma, and TFF1 may not interact or cooperate with GKN2. GKN2 overexpression can inhibit the growth and metastasis by downregulating the JAK2/STAT3 pathway in gastric cancer cells.

## 1. Introduction

Gastric cancer (GC) not only has a high incidence in the population of our country but also ranks high in mortality among many cancers [1]. The development of gastric cancer is a complex process of multistage and multistep. In this process, there are many genes involved, including the regulation of cell proliferation, apoptosis, differentiation, invasion, and metastasis. However, there are few molecules specifically expressed in gastric mucosa. GKN is a new family of gastrin-specific proteins, which is almost completely expressed and secreted by gastric mucosal epithelial cells. GKNs gene family is considered as a specific tumor suppressor gene of gastrointestinal tissue [2–4]. According to reports, GKN1 can inhibit the metastasis of gastric cancer cells and reduce their migration and invasion ability [5]. In gastric cancer, GKN2 (gastrokine-2) also has the same effect as GKN [6–9]. GKN2 is downregulation or loss in gastric cancer tissues. GKN2 is an obviously expressed gene after the elimination of *Helicobacter pylori* [10]. It shows that the regulatory pattern to cytokines is the same as those of the TFF gene [11]. It is reported that GKN2 affects the growth of gastric cancer cells in a trefoil factor 1- (TFF1-) dependent manner [12]. GKN2 forms disulfide-linked heterodimers with TFF1 [13, 14].

Although the downregulation of GKN2 expression in gastric cancer has been reported [15], the potential relationship between GKN2 and TFF1 in regulating the progression of gastric cancer and improving the biological behavior of cells remains unclear. The role of JAK2/STAT3 pathway in tumors is gradually discovered, and it also has a certain impact on the occurrence and development of gastric cancer [16–18]. In this study, we refer to the method in the previous study such as by Ling et al. [19]. We first examine the expressions of GKN2 and TFF1 in gastric cancer tissues, adjacent gastric mucosa, and distal gastric mucosa tissues using tissue chip and analyze its role in gastric carcinogenesis. Then, the constructed GKN2 expression vector was transfected into human gastric cancer MKN28 cells, and a stable transfection cell line was established. The proliferation, invasion, and migration of the cells were analyzed in order to explain the inhibitory effect of GKN2 on the growth of human gastric cancer MKN28 and SGC7901 cells through inhibiting the activation of the JAK2/STAT3 pathway. This study provides a good basis for the further study of the function of GKN2 in gastric cancer.

## 2. Materials and Methods

### 2.1. Experimental Method

#### 2.1.1. Materials

Gastric cancer tissue microarrays including 90 gastric cancers, 48 neoplastic resection margins, and 22 normal gastric mucosa epithelium >5 cm from the tumor edge were provided by the Department of Pathology, First Affiliated Hospital of University of South China. Clinicopathological data include tumor stage, degree of differentiation, age range, and gender. The study was approved by the Clinical review Committee of First Affiliated Hospital of University of South China.

Matrigel was provided by BD Company. Transwell chambers (8 *μ*m; Corning) were provided by Corning. MTT was provided by Beijing Kangwei Century Co., Ltd., China. The Ad-GFP-GKN2 expression vector and Ad-GFP-empty vector were constructed by Han Heng Biotechnology Co., Ltd. (Shanghai, China).

#### 2.1.2. Immunohistochemistry

The 4 *μ*m paraffin-embedded tissue sections were immunostained with citrate buffer antigen extraction and the UltrasensitiveTM SP streptavidin peroxidase signal amplification detection system (catalog number KIT-9710, Maixin Biotech. Co., Ltd. Fuzhou, China). The primary antisera were diluted 1 : 2000. The monoclonal anti-pS2 antibody (catalog number ab92377, Abcam, Carlsbad, CA) and the monoclonal anti-GKN2 antibody (catalog number ab184163, Abcam, Carlsbad, CA) were at a dilution of 1 : 50. DAB dye, hematoxylin staining, and neutral gum sealing slices were done. Criteria: the positive staining cells were found to be yellow or brown colored in the cytoplasm of the cells in the tissue microarray. The results were as follows: the number of stained cells less than 5 was negative in each high-power microscope. The number of stained cells more than 5 was positive in each high-power microscope.

#### 2.1.3. Cell Culture and Establishment of GKN2 Overexpressing Cell Lines

Human gastric cancer cell lines MKN28 and SGC7901 (Shanghai Gefan Biological Co., Ltd.) were preserved from our institute. Cells were stored in the RPMI1640 complete medium (Hangzhou Sijiqing Technology Co., Ltd., China), supplemented with 10% fetal bovine serum and placed in an incubator at 37°C and 5% CO_2_. MKN28 and SGC7901 cells were transfected with the Ad-GFP-GKN2 vector and Ad-GFP-empty vector. Blank, cells without any treatment; NC, negative control, cells transfected with Ad-GFP-empty vector negative control; GKN2, cells transfected with Ad-GFP-GKN2.

#### 2.1.4. qRT-PCR

Total RNA was extracted from cells or tissues using Trizol (catalog number 15596-018, Invitrogen), reverse transcribed to generate cDNA, and then, primers were amplified. Gene primers were synthesized by Invitrogen, as given in Table 1. *β*-Actin was used as a control for detecting the target gene. 2^−ΔΔCt^ was used to calculate the relative expression of the detected gene.

#### 2.1.5. CCK-8 Experiment

4 × 10^3^ cells were seeded in a 96-well plate, and a medium containing CCK-8 was added. CCK-8 accounted for 1/10 of the volume of the cell culture medium. After the color of the culture medium changes, took out the 96-well plate and put it into a microplate reader for detection and set the wavelength to 570 nm.

#### 2.1.6. Transwell Experiment

Cell migration was guided as previously described [7]. Briefly, MKN28 and SGC7901 cells were added to the upper chamber of the transwell chamber. The lower chamber was a culture medium containing 50 mg/L VEGF. After 1 day, it was rinsed with PBS, and 1 mL 4% paraformaldehyde was added to the lower chamber for fixation. 30 min, after proper drying, Giemsa staining for 30 min, rinsed with PBS, took out the filter cover, and 5 fields of view were randomly selected for counting. Cell invasion: MKN28 and SGC7901 cells were inoculated onto the Matrigel-coated filters. The cells were GKN2-transfected and untransfected for 24 h. Random use of hematoxylin staining is done. Invasion rates were represented as ratios between GKN2-transfected and control group values.

#### 2.1.7. Western Blot Analysis

Total protein was then extracted and quantified with a BCA protein assay kit. The total protein was separated by SDS-PAGE and transferred to the solid phase carrier. Anti-GKN2 (LSBio, 1 : 1000), anti-JAK2 (Abcam, 1 : 1000), anti-p-JAK2 (MilliporeSigma, 1 : 1000), anti-STAT3 (Abcam, 1 : 1000), anti-p-STAT3 (Cell Signaling Technology, 1 : 1000), and anti-*β*-actin (Santa Cruz Biotechnology, 1 : 1000) were added and incubated overnight at 4°C. *β*-Actin is an internal control. After washing and removing the unbound primary antibody, the NC membrane treated with the primary antibody is treated with the labeled secondary antibody for 1 hour. After the treatment is completed, wash 3 times, 10 minutes each time. Then, use a chemiluminescence kit to develop and evaluate the OD of the band density.

### 2.2. Statistical Analysis

Statistical analysis was carried out using the SPSS 18.0 program. The relevant row analysis of the categorical data was evaluated using the chi-square test. *P* < 0.05 was considered statistically significant. Associations between GKN2 and TFF1 expressions and the tumor histological type were tested using the Spearman test. Spearman rank correlation coefficient *r*_*s*_ is between −1 and 1, *r*_*s*_ < 0 as the negative correlation, and *r*_*s*_ > 0 as positive correlation.

## 3. Results

### 3.1. Expression of GKN2 and TFF1 in Gastric Carcinoma Tissues

GKN1 and TFF1 were highly expressed in distal gastric mucosa (DGM) but less in paracancerous tissue (PT). GKN2 and TFF1 staining are as shown in Figures 1(a)–1(d). Compared with the intestinal metaplasia area, the expression of GKN2 and TFF1 protein in gastric cancer was reduced (Figures 1(e)–1(h)).

Overall GKN2 expression was positive in 6.67% and negative in 78% of cancers (*p* < 0.05, *χ*2 = 11.19, or *χ*2 = 27.35), and TFF1 was lost in 78.89% of cancers (*p* < 0.05, *χ*2 = 29.45, or *χ*2 = 23.42), comparing with distal gastric mucosa (normal gastric mucosa epithelium) or paracancerous tissue (intestinal metaplasia) as given in Table 2.

### 3.2. Association between Expression of GKN2 and TFF1 in Gastric Carcinoma Tissues

It showed that six cases of GKN2 protein-positive expression include three cases of TFF1-positive expression in gastric cancer specimens, while 71 cases of TFF1-negative expression exist concurrently with 68 cases of GKN2-negative expression, namely, TFF1 protein expression loss is related to GKN2 protein expression loss as given in Table 3. The relationship between the two protein expressions seems to be a positive correlation (*r* ≈ ≈0.96), but statistics analysis showed the difference is meaningless (*p*=0.074).

### 3.3. Effect of GKN2 Overexpression on Proliferation of Human Gastric Cancer MKN28 and SGC7901 Cells

This study found that the Ad-GFP-GKN2 expression vector increased the expression of GKN2 mRNA in MKN28 and SGC7901 cells (*p* < 0.05, Figure 2(a)). Western blot detection also indicated that the GKN2 protein level of cells transfected with the Ad-GFP-GKN2 expression vector was significantly higher than that of the NC or blank group (*p* < 0.05, Figures 2(b) and 2(c)).

As shown in Figures 2(d) and 2(e), the proliferation of human gastric cancer MKN28 and SGC7901 cells in the GKN2 transfection group, NC, or blank group was observed. It indicated that the cell survival rate (OD570) of the transfected GKN2 cells decreased after transfection for 24 h, 48 h, and 72 h, compared with the NC and blank group.

### 3.4. Role of GKN2 Overexpression on Cell Migration and Invasion in MKN28 and SGC7901 Cells

The number of cells was observed and calculated migrating from the upper serum-free medium of the transwell chamber through the polycarbonate membrane to the lower serum-containing medium under the microscope. The cells are stained purple as shown in Figures 3(a) and 3(b). The number of cancer cells passing through the membrane in the GKN2 transfection group (26 ± 5) significantly lowered than that in the NC group (109 ± 7) and that in the blank group (110 ± 4) (*p* < 0.05).

As shown in Figures 3(c) and 3(d), GKN2 overexpression markedly decreased the number of MKN28 cells (28 ± 4) passing through Matrigel-coated membrane, compared with the NC group (67 ± 5) and blank group (66 ± 5) (*p* < 0.05).

### 3.5. GKN2 Knockin Inhibits the Activation of the JAK2/STAT3 Pathway in Gastric Cancer

As the Western blot results indicate, GKN2 overexpression markedly downregulated the expression of total JAK2, STAT3, and the level of the phosphorylated forms p-JAK2 and p-STAT3 in MKN28 and SGC7901 cells (*p* < 0.05, Figures 4(a) and 4(b)).

## 4. Discussion

GKN is a small protein in the BRICHOS superfamily [20, 21]. It has a domain of about 100 amino acids and is associated with inflammatory diseases, dementia, and cancer [22–24]. GKN2 is a protein specifically expressed in gastric mucosal epithelial cells, which may be a candidate tumor suppressor gene for gastric cancer [25]. It has been reported that GKN2 with biological activity can constantly regulate gastric mucosal immunity, inhibit tumor cell growth, inhibit EMT, metastasis, and invasion, that is, it can be used as a specific gastric tumor suppressor gene [26]. In normal human stomach, GKN2 showed endogenous overexpression, but miraculously, during the period from Hp infection to tumor formation, GKN2 showed a gradual downregulation, which was found in the study of human gastric tissue microarray. After the eradication of chronic *Helicobacter pylori* (Hp) infection, the upregulation of GKN2 gene was the most obvious among all the upregulated genes [10, 27]. With the increase of proinflammatory in the body, the expression of GKN2 gene also gradually decreases [28]. However, due to the difference between the tumor growth environment in vivo and in vitro cell culture environment, the expression of GKN2 in gastric cancer tissues, adjacent tissues, and normal gastric mucosa was analyzed. It was found that the expression of GKN2 was significantly higher in paracancerous tissue and distal gastric mucosa, but the expression was significantly lower in gastric cancer tissue than that in paracancerous tissue and distal gastric mucosa, indicating that GKN2 might play a role as a candidate tumor suppressor gene in gastric carcinogenesis and thus downregulate expression in gastric cancer. The downregulation of GKN2 in gastric cancer affects the prognosis of patients [29].

TFF is associated with mucous secreting epithelial cells. When the mucosa is invaded by bacteria, viruses, or drugs, inflammatory and ulcerative diseases occur, and they play a role in the recovery and regeneration of epithelial cells. TFF1 may act as a tumor suppressor gene in gastric cancer [30, 31], esophageal squamous cell carcinoma [32], and retinoblastoma [33], while it has been found to be overexpressed in colorectal cancer [34] and breast cancer [35]. Low expression of TFF1 may be a marker of poor prognosis in patients with early gastric cancer [36]. In vitro TFF1 can inhibit proliferation and induce apoptosis of cells [37, 38]. GKN2 has an unpaired cysteine residue, often forming a heterogeneous dimer with TFF1, secreted into the deep mucous layer, covering and protecting the underlying gastric epithelium [25]. Studies have found that GKN2 often forms a heterodimer in the form of disulfide bond with TFF1 of the clover protein family in the process of playing biological functions, and the two interact to play an antitumor role [39]. Studies have shown that GKN2 may play an inhibitory role in gastric cancer by coworking with TFF1 molecules [12]. We detected the expression of TFF1 in gastric cancer tissues, paracancerous tissues, and distal gastric mucosa. The results showed that the expression of TFF1 was positive in the distal gastric mucosa and paracancerous tissues, but significantly downregulated in gastric cancer tissues. It suggests that TFF1 may also be involved in the development of gastric cancer. What is more, studies have found gastric cancer with no GKN2 expression but TFF1 expression has a worse prognosis [14].

GKN2 can specifically interact with TFF1 [25, 40]. We analyzed the correlation between the expression of GKN2 and TFF in gastric cancer tissues. Our research proves that the expression of GKN2 and TFF1 is often downregulated in gastric cancer. It showed that half of the samples with positive expression of GKN2 protein were also positive for TFF1 [41]. However, GKN2 protein was not expressed in most of the specimens without TFF1 protein expression, and the expression of the two proteins showed a significant positive correlation, but there was no significant difference by statistical analysis, suggesting that the two proteins may not play a joint role in the carcinogenesis of gastric cancer. GKN2 may play an important role in gastric carcinogenesis through other pathways unrelated to TFF1, and its mechanism needs further study.

Studies have shown that GKN2 expression is downregulated or absent in gastric cancer cell lines [15]. GKN2 could control cell proliferation, migration, and invasion in gastric cancer cell line SGC7901 [15]. In the present study, the constructed GKN2 gene expression vector was transfected into human gastric cancer MKN28 cells, and it was found that overexpression of GKN2 could inhibit cancer cell proliferation, migration, and invasion. It is reported that some researchers have used bioinformatics and in vitro experiments to identify the functional DNA response elements of the STAT3 (SRE) signaling system in the 1 Kb sequence within the 20 Kb region of the GKN2 gene, and the STAT3 signaling pathway is one of the key components in the regulation of the GKN2 transcription level [42]. GKN2 gene is regulated by transcription factors such as STAT3 [43]. Therefore, the phenotype of GKN2 gene inhibiting proliferation is probably related to STAT3 or through the same signal transduction pathway. As everyone knows, activation of the JAK2/STAT3 pathway correlates with gastric cancer progression. The JAK2/STAT3 pathway has been found to be related to the migration and invasion of gastric cancer cells [44–46]. Therefore, the JAK2/STAT3 pathway may be able to evaluate the mechanism of GKN2 damage to gastric cancer cell metastasis. The study also found that the upregulation of GKN2 reduced the phosphorylation of JAK2 and STAT3 to achieve the purpose of inhibiting the JAK2/STAT3 pathway. The results suggest that GKN2 may participate in the influence on the growth and metastasis of gastric cancer cells by regulating the JAK2/STAT3 pathway. Based on the above results, we believe that GKN2 is a potential tumor suppressor gene in gastric cancer, and restoring the expression of GKN2 may be a new method for the treatment of gastric cancer. The study of the mechanism of GKN 2 is expected to further elucidate the pathogenesis of gastric cancer and provide the basis for finding a molecular target for the prevention and treatment of gastric cancer.

## 5. Conclusion

In summary, our research shows that GKN2 has an inhibitory effect on human gastric cancer, and GKN2 may play an antigastric effect by regulating the JAK2/STAT3 pathway. We believe that GKN2 may be a potential gastric cancer antitumor gene, and the GKN2/JAK2/STAT3 pathway may be a new target for the treatment of gastric cancer.

## Figures and Tables

**Figure 1:** Immunohistochemical staining of GKN2 and TFF1 expression in gastric tissues. Expression of GKN2 (a, c, e, g) and TFF1 (b, d, f, h). (a), (b) DGM; (c), (d) PT; (e), (f) GC (well-differentiated); (g), (h) GC (poorly differentiated). All original magnifications × 400. GKN2, gastrokine 2; TFF1, trefoil factor family 1; GC, gastric cancer; DGM, distal gastric mucosa; PT, paracancerous tissue.

**Figure 2:** GKN2 upregulation reduces proliferation of gastric cancer cells. (a) Expression of GKN2 mRNA in MNK28 and SGC7901 cells. (b), (c) Expression of GKN2 protein in MKN28 and SGC7901 cells. (d), (e) Cell proliferation of MKN28 and SGC7901 cells. ^*∗*^*P* < 0.05 vs. blank group. GKN2, gastrokine 2. NC, normal control.

**Figure 3:** GKN2 upregulation inhibits cell migration and invasion of gastric cancer cells. (a), (b) Cell migration of MKN28 and SGC7901 cells. (c), (d) Cell invasion of MKN28 and SGC7901 cells. All original magnifications × 400. ^*∗*^*P* < 0.05 vs. blank group. GKN2, gastrokine 2. NC, normal control.

**Figure 4:** GKN2 upregulation inhibits the activation of the JAK/STAT3 pathway. (a) Proteins in the JAK/STAT3 pathway in MKN28 cells. (b) Proteins in the JAK/STAT3 pathway in SGC7901 cells. ^*∗*^*P* < 0.05 vs. blank group. GKN2, gastrokine 2. NC, normal control.

**Table 1:** qRT-PCR primers.

Primer sequence	Forward (5′–3′)	Reverse (5′–3′)
GKN2	CTATGAGAAACAGGCTCTGG	TTGATCAGAGACTCCAGAGG
*β*-Actin	ACACTGTGCCCATCTACGAGGGG	ATGATGGAGTTGAAGGTAGTTTCGTGGAT

**Table 2:** GKN2 and TFF1 expressions in gastric tissues by immunohistochemical staining.

	Histological type	Positive	Negative	Number	Positive staining rate (%)
GKN2	DGM	19	3	22	83.36
	PT	21	27	48	43.75
	GC	6	84	90	6.67^*∗*^

TFF1	DGM	18	4	22	81.82
	PT	30	18	48	62.50
	GC	19	71	90	21.11^*∗*^

*Note*. ^*∗*^*P* < 0.05 vs. DGM. GKN2, gastrokine 2; TFF1, trefoil factor family 1; GC, gastric cancer; DGM, distal gastric mucosa; PT, paracancerous tissue.

**Table 3:** Correlation between GKN2 and TFF1 expression.

Group		TFF1	
		Positive	Negative
GKN2	Positive	3	3
	Negative	16	68

*Note*. GKN2, gastrokine 2; TFF1, trefoil factor family 1.

## Data Availability

The results are supported by data from Key Laboratory of Tumor Cellular and Molecular Pathology (University of South China), College of Hunan Province, Cancer Research Institute, Hengyang Medical College, University of South China.
